The article "Analysis of Risk Factors of Coagulation Dysfunction and Hemorrhage in Newly Diagnosed Hyperleukocytic Acute Myeloma Leukemia" was published in 2022. Journal: Contrast Media Mol Imaging.

# Analysis of Risk Factors of Coagulation Dysfunction and Hemorrhage in Newly Diagnosed Hyperleukocytic Acute Myeloma Leukemia

**DOI:** 10.1155/2022/7828230

**Published:** 2022-07-13

**Authors:** Anjie Xu, Pan Liu, Fuling Zhou

**Affiliations:** ^1^Second Clinical Medical College, Wuhan University, Wuhan, Hubei 430071, China; ^2^Department of Hematology, Xianning City Central Hospital, Xianning, Hubei 437000, China; ^3^Department of Hematology, Zhongnan Hospital of Wuhan University, Wuhan, Hubei 430071, China

## Abstract

**Purpose:**

To explore whether and why abnormal coagulation function and hemorrhage can appear in patients with hyperleukocytic acute myeloid leukemia (HAML).

**Method:**

We retrospectively reviewed the charts of 724 acute myeloid leukemia (AML) patients admitted with a white blood cell count of >100 × 10^9^/L between 2010 and 2019 in order to analyze the coagulation index of patients with HAML and explore the correlation of abnormal coagulation.

**Result:**

Prothrombin time (PT) was extended in group HAML compared with group non-HAML. Respiratory failure, intracranial hemorrhage, and infection were more common in the HAML group. Among the 76 HAML patients, there were 33 patients who had ≥3 abnormal items of coagulation index, and 51.5% of them had level 2 hemorrhage which was more than level 0 hemorrhage, and the difference is statistically significant (*P* < 0.01). Similarly, we can discover that 40.9% of patients with 2 abnormal items had level 2 hemorrhage in contrast to 0 abnormal items. The use of hydroxyurea had a significant effect on PT and D-dimer (DD). Survival analysis by the Kaplan–Meier method showed that there were statistically significant differences in white blood cell (WBC) count＞200 × 10^9^//L and DD. Abnormal PT is associated with WBC count＞200 × 10^9^//L, and abnormal activated partial thromboplastin time (APTT) is associated with HLA-DR mutation. Infection and respiratory failure were independent influencing factors for the coagulation of patients.

**Conclusion:**

DD had a marked effect on the survival rate. Infection and respiratory failure were independent influencing factors for the coagulation of patients.

## 1. Introduction

Hyperleukocytic acute myeloma leukemia (HAML) is one of the high-risk types and is defined as peripheral blood leukocyte counts exceeding 100 × 10^9^/L [1, 2]. Patients with acute myeloid leukemia (AML), especially those with HAML, are at an increased risk of early death and relapse [3]. HAML accounts for 10%–13% of the total AML and 7.3–8.5% of acute leukemia [4], and M2 and M5 are the most common types [5]. Without aggressive treatment, the 1-week fatality rate can be up to 40% [6]. HAML is a dangerous condition characterized by the excessive accumulation of white blood cells in blood vessels, tissues, and organs. Due to the high white blood cell count, it is prone to hyperviscosity and tumor lysis syndrome during chemotherapy and has a high early clinical mortality [7]. Hypercoagulability is one of the important pathogeneses of thrombosis or hemorrhage in patients. Besides, leukocytosis is a poorly understood and life-threatening complication in acute leukemia, which is associated with pulmonary congestion and infection, intracranial hemorrhage or infarction, melena, hematuria, and other complications [1, 8]. The pathogenesis may be that hyperleucocytes may increase extramedullary infiltration, enlarge lymph nodes, and aggravate liver and kidney injury [9]. In addition, leukemia can cause other complications by damaging the walls of small blood vessels and causing tissue bleeding. White blood cell (WBC) stasis in the lungs can affect blood flow, increase the hydrostatic pressure of pulmonary blood vessels, and increase exudate, which can lead to severe consequences such as acute respiratory distress syndrome (ARDS). The main types are AML and acute lymphocytic leukemia (ALL), and AML is the main one. Patients have extramedullary infiltration, disseminated intravascular coagulation (DIC), gastrointestinal bleeding, and other manifestations, and the onset is urgent. At present, it is not clear why HAML patients were prone to hemorrhage and whether there exists a relationship between coagulation function and hemorrhage, prognosis, gene mutation, immune, and cytogenic classification.

Therefore, it is very important to explore the early causes of hemorrhage and death in HAML patients and analyze their potential related risk factors for further improving the survival rate of HAML patients. In our retrospective study, we first analyzed the coagulation and hemorrhage of HAML and identified the risk factors associated with coagulation function.

## 2. Method

### 2.1. Patients

A total of 724 newly diagnosed AML patients at Wuhan University Zhongnan Hospital from January 2010 to December 2019 were collected from their medical records. Relapse, OS (overall survival), and CR (complete remission) were defined according to previously published criteria. All patients have signed informed consent forms and submitted them to Zhongnan Hospital for safekeeping. This study has been identified as fully consistent with the Declaration of Helsinki.

Patients were divided into the HAML group and non-HAML groups according to whether the leucocyte count was greater than 100 × 10^9^/L on admission. In the HAML group, the patients were selected into different levels of hemorrhage group according to clinical hemorrhage: Level 0: no symptoms of bleeding; Level 1: there are skin bleeding points, mild gingival or nasal bleeding, positive erythrocyte by uroscopy, positive occult fecal blood; Level 2: large skin ecchymosis and bleeding at injection site, nonstop bleeding from gums and/or nose, gross hematuria, black stool, fundus hemorrhage, and intracranial hemorrhage.

### 2.2. Experimental Data

The coagulation method was used for the determination of prothrombin time (PT), activated partial thromboplastin time (APTT), and thrombin time (TT). The thrombin method was used for the determination of fibrinogen (FIB), and the immunoturbidimetry method was used for determination of D-dimer (DD). The instruments were mainly from USES Ca-6000, a Sysmex automatic coagulation analyzer from East Asia, Japan, and Thermo Multiclan MK3, an enzyme marker analyzer from Finland.

### 2.3. Statistical Method

We used the SPSS Statistics 23 statistical analysis software. Overall survival and progression to AML were computed from the date of diagnosis. Patients were censored at the date of the last follow-up. The surviving data were described using the Kaplan–Meier method. Pearson and Spearman analysis was used to conduct a correlation analysis between abnormal coagulation indexes and tumor indexes. Single factor analysis was performed using the logistic analysis after preliminary rank test. All the results with *P* < 0.05 for the difference were statistically significant.

The PT reference range is 9.4∼12.5 s, the TT reference range is 12.3∼16.6 s, the APTT reference range is 25.1∼36.5 s, the FIB reference value is 238∼405 mg/mL, and the DD reference range is 0∼500 ng/mL. The patients' laboratory data were collected at or just after diagnosis.

## 3. Result

### 3.1. Study Population

In this study, we analyzed 724 patients who were diagnosed with AML from January 2010 to December 2019. The clinical and laboratory characteristics of the patients at the initial diagnosis are shown in Table 1. We found 76 patients with an initial leukocyte count greater than 100 × 109/L. There were 40 males and 36 females. The median age was 54 years (ranging from 17 to 80 years old). The median of leukocyte count on presentation was 181.890 × 109/L. Moreover, patients with HAML had thrombocytopenia but not below the lower limit.

At the presentation, PT extended and DD rose in group HAML compared with group non-HAML (*P* < 0.05). The poor cytogenetic prognosis rates in group HAML were lower than in non-HAML group (*P* < 0.05). Respiratory failure, intracranial hemorrhage, and infection were more common in the HAML group.

### 3.2. Hemorrhage Analysis

There were 76 hemorrhage patients in group HAML (Table 2). Among the 76 patients, there were 33 patients who had ≥3 abnormal items of the coagulation index, and 51.5% of them had level 2 hemorrhage, which was more than level 0 hemorrhage, and the difference was statistically significant (*P* < 0.01). Similarly, we can discover that 40.9% of patients with 2 abnormal items had level 2 hemorrhage in contrast to 0 abnormal items (*P* < 0.05).

### 3.3. Time Curve of Coagulation Function of Patients with HAML

According to different treatments, HAML patients were divided into two groups: the hydroxyurea group and the apheresis group. All patients received IA regimen chemotherapy (cytarabine + IDNR). As shown in Figure 1, by comparing the curves of coagulation function in average value over time in HAML patients, we found that PT and DD decreased after hydroxyurea and apheresis, and patients gradually changed from the risk state of high coagulation to the normal state. But in fact, there was no difference in the therapeutic effect between the hydroxyurea group and the apheresis group.

### 3.4. Survival Analysis

Survival analysis by the Kaplan–Meier method showed that there were statistically significant differences in WBC count ＞200 × 10^9^//L and DD (*P* < 0.05), as shown in Figure 2.

To assess the role of other clinical indicators of coagulation function in predicting outcome death, we performed a multivariate analysis using a Cox regression model in Table 3, and DD and WBC >200 × 10^9^//L are prognosis independent risk factors of HAML.

### 3.5. Correlation Analysis

According to the analysis of correlation analysis between abnormal coagulation indexes and tumor indexes in Table 4, abnormal DD is associated with infection, bleeding level, and OS (Table 4).

At the same time, logistic analysis was carried out to study the factors of abnormal coagulation indicators in HAML patients. The results showed that infection and respiratory failure were independent influencing factors for the coagulation of patients (Table 5).

### 3.6. Coagulation Function of HAML Patients with Infection and Respiratory Failure

According to the results of the Logistics analysis, we separately analyzed the coagulation function indicators of HAML patients with infection and respiratory failure. As shown in Figure 3, FIB and DD were elevated and there were significant differences in infected HAML patients. Furthermore, DD was elevated and significantly different in HAML patients with respiratory failure.

## 4. Discussion

Hyperleukocytosis has been suggested to be a risk factor for venous thrombosis in a variety of organs [8, 10–14]. Hyperleukocytic hemorrhage was considered to occur due to vascular rupturing caused by leukemic thrombi and/or necrosis of ischemic tissue [15, 16]. In the present study, HAML patients were more frequent in early death (within a week) and more likely to have bad gene mutations and poor cytogenetic prognosis. In our study population, abnormal coagulation function and increased WBC count greatly affected the overall survival (OS) of HAML patients.

Compared with non-HAML patients, HAML patients were more likely to have abnormal coagulation function and were more likely to be accompanied by hemorrhage complications, gene mutations, and chromosomal karyotypes with poor prognoses. Hemorrhage may occur in either acute lymphocytic leukemia (ALL) or AML [17–19]. The hemorrhages in HAML patients were associated with abnormal coagulation function in our present study.

There is a certain correlation between hemorrhage and coagulation dysfunction in HAML patients. The more severe the bleeding symptoms were, the more the coagulation dysfunction items were to be.

Abnormal coagulation function and increased WBC count greatly affected the survival rate of HAML patients.

Finally, we found that infection and respiratory failure were the factors influencing coagulation dysfunction. Patients with HAML had abnormal PT, which was related to the WBC count. PT is the main reflection of exogenous blood coagulation. Therefore, we hypothesize that the coagulation abnormalities in patients with HAML are mainly related to exogenous coagulation dysfunction. We further hypothesize that factors such as respiratory failure in patients with HAML elevated coagulation factor III, leading to exogenous coagulation dysfunction [20], but the conjecture needs further verification.

Bleeding occurs mainly when the white blood cell count is extremely high, and causes include increased blood viscosity and reduced ability to burst and deform. Histopathological findings suggest that the bleeding complication may be due to bleeding following the initial leukocyte thrombosis. The aggregation of leukocyte thrombi may be caused by the upregulation of specific adhesion molecules induced by leukemic cells. In addition, sequential leukocytosis, pulmonary, cardiac or cerebrovascular obstruction, hemorrhage, and edema are suggested [21]. Endothelial damage is also thought to be a trigger for coagulation abnormalities [22, 23].

Although some studies have found that leukapheresis was useful for reducing the early mortality rate and preventing hemorrhage in AML patients with hyperleukocytosis [3], it has been reported that leukapheresis did not improve survival or decrease the incidence of hemorrhage in adults with HAML. Furthermore, the latter study demonstrated that early chemotherapy (within 48 h of admission) resulted in better outcomes than delayed chemotherapy in terms of the risk of early death [11]. Recently, it was reported that leukapheresis and low-dose chemotherapy did not reduce early mortality in AML patients with hyperleukocytosis in a meta-analysis [15]. But other research has shown that leukapheresis reduces 4-week mortality in AML patients with hyperleukocytosis [24].

It was also reported that a large number of hyperleukocytic AML patients who underwent leukapheresis showed a significant decrease in fibrinogen and a significant increase in PT, INR, and DIC scores after the procedures [25]. In our study, the use of hydroxyurea and apheresis had a significant effect on DD and PT. Besides, the efficacy of hydroxyurea and apheresis was similar, and patients gradually returned to their normal state.

Although the pathogenesis of acute leukemic leukemia is actively explored and the tumor burden of leukemia is reduced as much as possible, the progression of acute leukemic leukemia is still fast. More clinical studies are needed to provide evidence for the control of the disease development so as to reduce the early mortality, gain more opportunities for chemotherapy or transplantation, and delay the survival time.

## 5. Conclusion

The occurrence of abnormal coagulation index was a significant affecting factor for HAML in patients, and DD had a marked effect on survival rate. Infection and respiratory failure were independent influencing factors for the coagulation of patients. In addition, patients with HAML commonly accompanied with abnormal coagulation are exposed to a high risk of hemorrhage. HAML patients with respiratory failure and infection are more likely to have abnormal coagulation.

## Figures and Tables

**Figure 1:** Time curve of coagulation function of patients with HAML. PT: prothrombin time; FIB: the fibrinogen; APTT: activated partial thromboplastin time; DD: D-dimer.

**Figure 2:** K-M survival curve of patients with hyperleukocytosis. WBC: white blood cell; DD: D-dimer; *P* values were calculated using the univariate proportional-hazard model.

**Figure 3:** Coagulation function of HAML patients with infection (a) and respiratory failure (b) RF: respiratory failure.

**Table 1:** Analysis on the basic features and coagulation index of HAML and non-HAML patients.

	HAML (*n* = 76)	Non-HAML (*n* = 648)	*P* value
Clinical characteristics			
Sex (*n*)			
Male	40	410	0.049
Female	36	238	
Age (mean)	54	47	0.193
WBC (×10^9^//L)	181.890 ± 92.15	21.221 ± 15.971	＜0.005
PLT (×10^9^//L)	60.07 ± 71.101	63.97 ± 73.324	＜0.005
HGB (g/L)	72.730 ± 26.342	77.800 ± 25.342	0.164
RBC (×10^12^//L)	2.300 ± 1.033	3.261 ± 11.937	0.5115
Coagulation index			
PT (s)	17.133 ± 12.860	14.100 ± 8.940	＜0.005
FIB (mg/dL)	322.741 ± 118.92	340.147 ± 171.510	＜0.005
APTT (s)	34.139 ± 12.74	33.610 ± 6.101	0.721
DD (ng/mL)	3849.276 ± 6742.661	1329.32 ± 1811.171	＜0.005
TT (s)	13.291 ± 13.782	14.052 ± 9.460	0.579
Immune classification			
CD117+	32.8%	19.7%	＜0.005
CD13+	21.3%	20.8%	0.312
HLADR	23.1%	22.1%	0.479
CD38+	17.9%	18.2%	0.092
Gene mutation			
FLT3-ITD	24.3%	19.1%	＜0.005
CEBPA	8.1%	11.6%	＜0.005
C-kit/D816	9.2%	9.4%	0.213
Cytogenetic prognosis			
Good	7.9%	9.5%	0.1893
Poor	19.2%	7.0%	＜0.005
Complication			
Respiratory failure	33.3%	23.6%	＜0.005
Intracranial hemorrhage	64,1%	33.0%	＜0.005
Heart failure	19.2%	18.7%	0.942
Infection	71.8%	67.5%	＜0.005

HAML: hyperleukocytic acute myeloma leukemia; WBC: white blood cell; PLT: platelet; Hb: hemoglobin; PT: prothrombin time; FIB: fibrinogen; APTT: activated partial thromboplastin time; DD: D-dimer; TT: thrombin time; *P* values were calculated using the univariate Cox proportional-hazard model.

**Table 2:** Abnormal rates of coagulation indexes and hemorrhage rates in 76 patients with hyperleukocytic.

Abnormal items of coagulation index	*n*	Level 0 hemorrhage	Level 1 hemorrhage	Level 2 hemorrhage
0 items	6	6 (100%)	0 (0%)	0 (0%)
1 item	15	5 (33.3%)	6 (40%)	4 (26.7%)
2 items	22	3 (13.6%)	10 (45.5%)	9 (40.9%)^*∗*^
≥3 items	33	6 (18.2%)	10 (30.3%)	17 (51.5%)^*∗∗*^

Level 0: no symptoms of bleeding; Level 1: there are skin bleeding points, mild gingival or nasal bleeding, positive erythrocyte by uroscopy, positive occult fecal blood; Level 2: large skin ecchymosis and bleeding at the injection site, nonstop bleeding from gums and/or nose, gross hematuria, black stool, fundus hemorrhage, intracranial hemorrhage. Compared with 0 abnormalities, ^*∗*^*P* < 0.05; compared with 0 items, ^*∗∗*^*P* < 0.01.

**Table 3:** Survival Cox analysis of regression.

	Wald	B	Exp (B)	S.E.	Sig.
DD	5.019	0.01	1.211	0.005	0.024^*∗∗*^
WBC >200 × 10^9^//L	7.089	0.004	1.104	0.829	0.008^*∗∗∗*^
Age	9.474	0.029	1.03	0.009	0.2
Heart failure	11.827	1.661	1.190	0.483	0.190
PLT (×10^9^//L)	5.102	0.01	0.932	0.005	0.581
PT	4.333	0.018	1.018	0.009	0.084
APTT	7.921	0.024	1.029	0.033	0.396
TT	13.751	0.236	1.022	0.002	0.627
FIB	9.231	0.012	1.012	0.079	0.094
CKMB	7.510	0.031	1.043	0.091	0.434
CD13+	8.232	0.038	0.945	0.341	0.934
CD117+	7.27	0.918	1.011	0.641	0.132
CD33+	6.69	0.024	1.036	0.669	0.413
Abnormal coagulation function indicators	6.969	0.401	1.494	0.152	0.08
WT1+	1.788	0.472	1.604	0.480	0.618
FLT3+	9.763	0.145	1.081	0.065	0.963
Apheresis	9.14	1.031	1.201	0.259	0.339
Hydroxycarbamide	8.64	0.017	1.086	0.031	0.079

^*∗*^ *P* < 0.05; ^*∗∗*^*P* < 0.01.

**Table 4:** Correlation Pearson analysis between abnormal coagulation indexes and tumor indexes.

		PT	APTT	DD	TT	FIB
Tumor burden	*R* value	0.038	0.461	0.084	0.185	0.063
	*P* value	0.858	0.211	0.580	0.229	0.591

WBC (×10^9^//L)	*R* value	0.027	0.029	0.032	0.096	0.117
	*P* value	0.858	0.802	0.785	0.443	0.233

CD117+	*R* value	0.110	0.130	0.102	0.316	0.092
	*P* value	0.548	0.478	0.577	0.089	0.193

CD33+	*R* value	0.055	0.065	0.01	0.015	0.035
	*P* value	0.768	0.725	0.985	0.935	0.297

CD13+	*R* value	0.131	0.184	0.004	0.095	0.096
	*P* value	0.492	0.330	0.984	0.623	0.133

Infection	*R* value	0.126	0.052	0.431	0.187	0.101
	*P* value	0.360	0.704	0.01^*∗∗∗*^	0.172	0.468

Bleeding level	*R* value	0.06	0.202	0.294	0.012	0.018
	*P* value	0.604	0.08	0.01^*∗∗*^	0.926	0.853

OS (days)	*R* value	0.104	0.065	−0.373	0.036	−0.123
	*P* value	0.423	0.611	0.001^*∗∗∗*^	0.791	0.274

Age	*R* value	0.103	0.15	0.128	0.066	0.125
	*P* value	0.374	0.226	0.270	0.598	0.202

^*∗∗*^ *P* ≤ 0.01,^*∗∗∗*^*P* ≤ 0.001.

**Table 5:** Logistics analysis of influencing factors for abnormal coagulation function (≥1 abnormal among 5 data items) in patients with HAML.

	Wald	Exp (B)	S.E.	95% CI	*P* value
FLT3-ITD	4.305	1.875	0.280	0.084–0.232	0.230
NPM1	0.967	0.619	0.829	0.619–5.516	0.631
CEBPA	6.069	1.833	0.733	0.323–10.407	0.089
PLT	0.155	1.014	0.035	0.947–1.086	0.693
Hb	0.220	0.995	0.011	0.975–1.016	0.501
Neutrophils	3.028	1.100	0.055	0.988–1.224	0.296
RBC	1.091	0.742	0.285	0.424–1.299	0.596
Sex	0.282	0.733	0.584	0.233–2.305	0.112
Age	2.530	1.026	0.016	0.994–1.020	0.752
HLA-DR+	0.625	2.412	1.113	2.471–21.378	0.722
CD13+	10.793	0.200	0.490	0.579–22.794	0.712
CD38+	4.236	5.136	0.795	0.22–4.931	0.117
CD33+	0.256	0.714	0.665	0.194–2.628	0.613
WBC >200 × 10^9^//L	0.057	1.158	0.613	0.348–3.847	0.811
Abnormal liver function	0.051	1.143	0.594	0.295–3.288	0.135
Abnormal renal function	0.010	0.984	0.615	0.991–1.001	0.831
FAB type	7.735	0.145	1.282	0.012–1.791	0.102
Infection	9.927	1.143	0.688	0.032–0.471	0.007^*∗∗∗*^
Tumor burden	0.049	1.003	0.015	0.974–1.033	0.825
Respiratory failure	9.650	1.667	0.614	0.015–0.498	0.008^*∗∗∗*^

^*∗*^ *P* < 0.05,^*∗∗∗*^*P* < 0.001.

## Data Availability

The datasets used and analyzed during the current study are available from the corresponding author upon reasonable request.
